The article "Erythropoietin Restores Long-Term Neurocognitive Function Involving Mechanisms of Neuronal Plasticity in a Model of Hyperoxia-Induced Preterm Brain Injury" was published in 2016. Journal: Oxid Med Cell Longev.

# Erythropoietin Restores Long-Term Neurocognitive Function Involving Mechanisms of Neuronal Plasticity in a Model of Hyperoxia-Induced Preterm Brain Injury

**DOI:** 10.1155/2016/9247493

**Published:** 2016-07-14

**Authors:** Daniela Hoeber, Marco Sifringer, Yohan van de Looij, Josephine Herz, Stéphane V. Sizonenko, Karina Kempe, Meray Serdar, Joanna Palasz, Martin Hadamitzky, Stefanie Endesfelder, Joachim Fandrey, Ursula Felderhoff-Müser, Ivo Bendix

**Affiliations:** ^1^Department of Paediatrics I, Neonatology, University Hospital Essen, University Duisburg-Essen, 45147 Essen, Germany; ^2^Institute of Physiology, University of Duisburg-Essen, 45147 Essen, Germany; ^3^Department of Anaesthesiology and Intensive Care Medicine, Charité-Universitätsmedizin Berlin, Campus Virchow-Klinikum, 13353 Berlin, Germany; ^4^Division of Child Growth and Development, Department of Paediatrics, University of Geneva, 1205 Geneva, Switzerland; ^5^Laboratory of Functional and Metabolic Imaging, Ecole Polytechnique Fédérale de Lausanne, 1015 Lausanne, Switzerland; ^6^Institute of Medical Psychology and Behavioral Immunobiology, University Hospital Essen, University Duisburg-Essen, 45147 Essen, Germany; ^7^Department of Neonatology, Charité-Universitätsmedizin Berlin, 13353 Berlin, Germany

## Abstract

Cerebral white and grey matter injury is the leading cause of an adverse neurodevelopmental outcome in prematurely born infants. High oxygen concentrations have been shown to contribute to the pathogenesis of neonatal brain damage. Here, we focused on motor-cognitive outcome up to the adolescent and adult age in an experimental model of preterm brain injury. In search of the putative mechanisms of action we evaluated oligodendrocyte degeneration, myelination, and modulation of synaptic plasticity-related molecules. A single dose of erythropoietin (20,000 IU/kg) at the onset of hyperoxia (24 hours, 80% oxygen) in 6-day-old Wistar rats improved long-lasting neurocognitive development up to the adolescent and adult stage. Analysis of white matter structures revealed a reduction of acute oligodendrocyte degeneration. However, erythropoietin did not influence hypomyelination occurring a few days after injury or long-term microstructural white matter abnormalities detected in adult animals. Erythropoietin administration reverted hyperoxia-induced reduction of neuronal plasticity-related mRNA expression up to four months after injury. Thus, our findings highlight the importance of erythropoietin as a neuroregenerative treatment option in neonatal brain injury, leading to improved memory function in adolescent and adult rats which may be linked to increased neuronal network connectivity.

The article "Erythropoietin Restores Long-Term Neurocognitive Function Involving Mechanisms of Neuronal Plasticity in a Model of Hyperoxia-Induced Preterm Brain Injury" was published in 2016. Journal: Oxid Med Cell Longev.

## 1. Introduction

Over the last 20 years considerable progress in the care of high-risk prematurely born infants has led to increased survival, but also to a change in the pattern of pathology associated with neurological impairments [1]. Cystic focal lesions leading to cerebral palsy are now less common [2, 3], but the predominant neuropathological hallmark is a more subtle and diffuse type of damage involving impaired development of grey and white matter [4]. Recent findings from clinical MRI studies at term equivalent age led to the assumption that adverse neurodevelopmental outcome is primarily attributed to disturbed glial maturation and neural connectivity rather than to cell death alone [5]. As a result, survivors of preterm birth suffer from altered function ranging from severe motor impairment to cognitive problems, attention deficit disorders, behavioural alterations, and psychiatric disease [6, 7]. The latter have brought the search for neuroprotective and/or regenerative therapies into the focus of preclinical experiments to prepare for clinical trials. Since preterm brain injury involves a complex pathophysiology with acute and chronic phases, preclinical testing of potential therapeutic compounds targeting multiple mechanisms of neural cell injury and maturation in adequate experimental models is highly warranted. Epidemiological studies revealed that exposure to high oxygen concentrations at atmospheric pressure is a contributor to a poor outcome in survivors of preterm birth [8, 9], leading to caution with the use of supplementary oxygen during the perinatal period [10]. Therefore a preterm rodent model of oxygen-induced brain damage has been developed mimicking the clinical situation [11, 12]. Hyperoxia-triggered subtle neurodegeneration in rodents is associated with inflammation, oxidative stress response, growth factor deficiency, and transient hypomyelination with long-lasting microstructural changes in the white matter [13–17]. Recent studies in rodents further revealed hyperactivity and coordination deficits at adolescent age [18] and cognitive impairment persisting into adulthood [19], which parallel the clinical situation in preterm infants.

Erythropoietin (Epo) is an endogenous 30.4 kDa protein which is in clinical use for years to prevent anaemia of prematurity [20]. Retrospective evaluation of several clinical trials primarily addressing stimulation of erythropoiesis suggested Epo as a potential therapeutic agent for neonatal brain injury [21]. Epo is produced in the developing brain by multiple cell types (neurons, oligodendrocytes, microglia, and astrocytes) and may act as a growth factor, providing endogenous neuroprotection upon an injurious stimulus [22, 23]. In the past the effects of Epo treatment have been studied in rodents and nonhuman primates in hypoxic-ischemic injury representing a model of term asphyxia and stroke and recently also in combination with therapeutic hypothermia [24–26]. Clinical trials are underway evaluating its safety and neuroprotective properties for term asphyxia, neonatal stroke, and congenital cyanotic heart disease and also include the preterm population [27]. However, very few experimental studies in the past focused on preterm models such as intrauterine hypoxia-ischemia [28, 29] and hypoxia-ischemia at postnatal day 3 (P3) [30]. Hardly any experimental model addressed subtle diffuse brain injury types such as perinatal inflammation or hyperoxia [31]. However, in the context of the use of Epo in oxygen-induced cerebral injury in rodents, modulation of inflammatory cascades, growth factor signalling, and autophagy activity have been shown besides its antiapoptotic and antioxidative capacities [16, 32–34]. Still, current knowledge of its impact on myelination, neuronal networks, and long-term functional outcome is limited.

The article "Erythropoietin Restores Long-Term Neurocognitive Function Involving Mechanisms of Neuronal Plasticity in a Model of Hyperoxia-Induced Preterm Brain Injury" was published in 2016. Journal: Oxid Med Cell Longev.

Our goal in the present study was to test the hypothesis that single intraperitoneal injection of high-dose Epo in 6-day-old rats attenuates the long-term consequences of experimental hyperoxia-induced brain injury. Therefore we investigated white matter injury and elucidated mechanisms involved in synaptogenesis and formation of neuronal networks up to adulthood. In addition, long-term neurobehavioural, motor, and cognitive testing was applied at adolescent and adult age.

## 2. Materials and Methods

### 2.1. Animals and Experimental Procedures

All animal experiments were approved and performed in accordance with the guidelines of the University Hospital Essen, Germany, and with permission of the local animal welfare committee.

6-day-old Wistar rat pups were placed together with their lactating dams in an oxygen chamber (OxyCycler, BioSpherix, Lacona, NY, USA) for 24 hours containing 80% oxygen (80%). Hyperoxic dams underwent treatment only once and control animals were kept under normoxic conditions at 21% oxygen (21%). Based on our previous work [33] animals received a single intraperitoneal (i.p.) dose of 20,000 IU/kg body weight of recombinant erythropoietin (Epo, NeoRecormon®, Boehringer-La Roche, Grenzach, Germany) or equal amounts of normal saline (10 mL/kg body weight) at the onset of hyperoxia, resulting in four study groups: normoxia + normal saline (21%), normoxia + Epo (21% + Epo), hyperoxia + normal saline (80%), and hyperoxia + Epo (80% + Epo). A total of 139 sex-matched rat pups were enrolled in the study and randomly assigned to the treatment groups with at least two litters per experiment and per analysis protocol to ensure heterogeneity. Bodyweight was recorded regularly and there were no significant changes in weight gain between experimental groups. For different analysis protocols, pups were sacrificed at postnatal day 7 (P7) (57 pups, 5 litters), P11 (36 pups, 3 litters), and P125 (44 pups, 4 litters) under deep anaesthesia. In accordance with our previous observations [11, 13, 19] acute and subacute white matter impairment with cellular oligodendrocyte degeneration and myelin basic protein (MBP) expression were determined at P7 and P11, respectively. Functional deficits and behavioural abnormalities were analysed at adolescent (P30) and adult (P90) developmental stage and the same animals were partially used for postmortem diffusion tensor imaging (DTI) performed at P125 to evaluate long-term microstructural white matter changes and mRNA analysis of neuroplasticity-associated genes. mRNA analysis was moreover conducted at P7 and p11 (latter animals also used for MBP protein analysis). For protein and mRNA analysis, rats were transcardially perfused with phosphate buffered saline (PBS) and brain hemispheres were snap-frozen in liquid nitrogen. For histological and DTI studies, pups were transcardially perfused with PBS followed by 4% paraformaldehyde (PFA, Sigma-Aldrich, Munich, Germany). Brains were postfixed in 4% PFA overnight at 4°C and embedded in paraffin or sent for diffusion tensor imaging.

The article "Erythropoietin Restores Long-Term Neurocognitive Function Involving Mechanisms of Neuronal Plasticity in a Model of Hyperoxia-Induced Preterm Brain Injury" was published in 2016. Journal: Oxid Med Cell Longev.

### 2.2. Behavioural Studies

Behavioural testing was initiated in adolescent animals from P30 to P38 and repeated from P90 to P98 in adulthood. From P20, animals were familiarised with the investigator through every-other-day-handling during the active phase under an inverse 12-hour light-dark cycle. Testing started with one day of open field followed by four days of novel object recognition and completed with four days of Barnes maze. To avoid intramaze cues due to odour, mazes were carefully cleaned after each animal. Data was recorded using an automatic tracking system (Video-Mot2, TSE Systems, Bad Homburg, Germany) and exported for statistical analysis.

For the open field test [35], animals were placed into the centre of a dimly lit open field arena (50 × 50 × 40 cm for adolescent or 75 × 75 × 40 cm for adult animals) placed upon an infrared-box (850 nm, TSE Systems). Movements were recorded by the tracking system for 10 minutes. General motor activity, that is, travelled distance and velocity, was analysed. The novel object recognition test was performed according to Chambon et al. with minor adaptations [36]. Animals were placed into the centre of a Y-maze (arm length: 60 cm; width: 26 cm; wall height: 56 cm) under red light. From inside the maze no external cues were visible. The first day, during habituation, animals were allowed to explore the empty arena. The next two days, three identical objects (white pyramids) were placed at the end of the maze arms for familiarisation. For the testing phase on day four, one of the familiar objects was replaced by a novel object consistent in height and biologically inert material but differently shaped (black cylinder). In each phase animals were exposed to the arena for five minutes and the time spent at each object was detected by the software. According to Chambon et al. analysis was performed for the first two minutes of testing time [36]. Spatiotemporal memory was assessed by the Barnes maze [37] as described previously [19]. Briefly, the animals were placed into the centre of the maze (1.22 m width, 0.8 m height, 20 holes at the border, TSE Systems) under red light followed by bright light to allow the animal to recognise extra-maze cues. The animals were allowed to explore the maze and find the escape box within 120 seconds; afterwards the animals were left in the escape box for 1 minute. Animals who did not find the escape box were gently placed into it for 1 minute. To avoid intramaze cues due to odour the escape box was rotated clockwise for every other animal, with the same escape location for each animal as on the three training days. The latency to find the trained escape box was assessed on the fourth day of each experiment when all holes were closed [38].

The article "Erythropoietin Restores Long-Term Neurocognitive Function Involving Mechanisms of Neuronal Plasticity in a Model of Hyperoxia-Induced Preterm Brain Injury" was published in 2016. Journal: Oxid Med Cell Longev.

### 2.3. Immunohistochemistry and Confocal Microscopy

After deparaffinisation, 10 *μ*m coronal sections (−3.72 ± 0.7 mm from bregma) were rehydrated. Antigen-retrieval was performed in a preheated 10 mM sodium-citrate buffer (pH 6.0) for 30 minutes. After blocking with 1% bovine serum albumin and 0.3% cold fish skin gelatin in 0.1% Tween-20 Tris-buffered saline (Sigma-Aldrich), all slides were incubated with primary antibodies overnight at 4°C followed by appropriate secondary antibody incubation for 1 hour at room temperature. Degeneration of oligodendrocytes was evaluated at P7 via colabelling with Olig2 (1 : 100, polyclonal rabbit anti-Olig2, Millipore, Darmstadt, Germany), followed by appropriate secondary antibody staining (1 : 300, anti-rabbit Alexa Fluor 594, Invitrogen, Karlsruhe, Germany) and terminal deoxynucleotidyl transferase-mediated dUTP nick end labelling (TUNEL, in situ cell death detection kit, FITC, Sigma-Aldrich), performed according to the manufacturer's instructions. Sections were counterstained with 4,6-diamidino-2-phenylindole (DAPI) (1 *μ*g/mL, Invitrogen, Karlsruhe, Germany). For exemplary image acquisition three laser lines (laser diode, 405 nm; Ar laser, 514 nm; G-HeNe laser, 543 nm) and three different filters (450/50-405 LP, 515/20-540 LP, and 585/65-640 LP) were used. Confocal z-stacks of 10 *μ*m thickness (z-plane distance 1 *μ*m) were converted into 2-dimensional images using maximum intensity projections. Analysis was performed by an observer blinded to treatment. Degenerating oligodendrocytes were analysed in 2 sections per animal by counting triple-positive (Olig2^+^/TUNEL^+^/DAPI^+^) cells, respectively, at 20x magnification under an inverted confocal fluorescence microscope system (A1 Eclipse Ti, Nikon, Düsseldorf, Germany). Oligodendrocyte degeneration was assessed in four different regions of interest: corpus callosum, deep cortical white matter, cortex, and thalamus. Data are expressed as the average of Olig2/TUNEL positive cells per mm^2^.

The article "Erythropoietin Restores Long-Term Neurocognitive Function Involving Mechanisms of Neuronal Plasticity in a Model of Hyperoxia-Induced Preterm Brain Injury" was published in 2016. Journal: Oxid Med Cell Longev.

### 2.4. Immunoblotting

Western blotting was performed with hemisphere protein lysates (40 *μ*g per sample) as described previously [13]. Membranes were incubated overnight at 4°C with a primary monoclonal mouse anti-MBP antibody (1 : 10,000, Abcam, Cambridge, UK) detecting two classical isoforms at 18.5 kDa and 21.5 kDa and with polyclonal rabbit anti-glyceraldehyde 3-phosphate dehydrogenase (GAPDH) antibody (37 kDa; 1 : 1000, Santa Cruz, Heidelberg, Germany). Membranes were incubated for 1 hour at room temperature with horseradish peroxidase-conjugated secondary anti-mouse (1 : 5000, Dako, Hamburg, Germany) or anti-rabbit (1 : 2000, Dako) antibody. All antibodies were diluted in 5% nonfat dry milk in Tris-buffered saline and 0.05% Tween-20 (Sigma-Aldrich). Antibody binding was detected by using enhanced chemiluminescence (GE Healthcare Life Sciences, Munich, Germany). For visualisation and densitometric analysis ChemiDoc XRS+ imaging system and ImageLab software (Bio-Rad, Munich, Germany) were used. Since several isoforms of MBP exist, the 21.5 kDa isoform known to be increased during early active myelination [39] was quantified. Data were expressed as density ratio of analysed protein/reference protein GAPDH with control group set to 1.

### 2.5. Diffusion Tensor Imaging

At P125,* ex vivo* brains from behaviour tested animals were subjected to diffusion tensor imaging. All experiments were performed on an actively shielded 9.4 T/31 cm magnet (Varian/Magnex Scientific, Oxford, UK) equipped with 12 cm gradient coils (400 mT/m, 120 *μ*s) with a transceiver 25 mm birdcage volume RF coil. First- and second-order shims were adjusted manually, with a water bandwidth ranging between 20 and 30 Hz. Diffusion gradients were applied along 6 spatial directions in a spin echo sequence [40]. The intensity (*G*_*d*_), duration (*δ*), and separation time of the pulsed diffusion gradients were set to 22 G/cm, 3 ms, and 20 ms, respectively (*b*-value of 1185 s/mm^2^). A field of view of 27 × 27 mm^2^ was sampled on a 128 × 128 Cartesian grid and 12 slices of 0.8 mm thickness were acquired in the axial plane with 20 averages. The echo time was set to 35 ms and the repetition time between consecutive measurements was 2000 ms. Using homemade Matlab (Mathworks, Natick, MA, USA) software, the radial diffusivity (*D*_⊥_), the axial diffusivity (*D*_//_), the mean diffusivity (MD), and the fractional anisotropy (FA) were derived from the tensor. The program allows manual delineation of region of interest (ROI) on the direction encoded colour maps. On two different structures of the brain (corpus callosum (CC) and external capsule (EC)), ROIs were carefully manually delimited at 6 different image-planes of the brain from the genu to the splenium of the corpus callosum.

The article "Erythropoietin Restores Long-Term Neurocognitive Function Involving Mechanisms of Neuronal Plasticity in a Model of Hyperoxia-Induced Preterm Brain Injury" was published in 2016. Journal: Oxid Med Cell Longev.

### 2.6. RNA Extraction and Semiquantitative Real-Time PCR

Total RNA was isolated from snap-frozen tissue by acidic phenol/chloroform extraction (peqGOLD RNAPure*™*; PEQLAB Biotechnologie, Erlangen, Germany) and 2 *μ*g of RNA was reverse transcribed. Gene expression analysis was performed as previously described using the PCR ABI Prism 7500 (Applied Biosystems, Foster City, CA, USA [13, 41]). The PCR products of* synaptophysin*,* neuregulin-1*,* neuropilin-1,* and*β-actin* (as internal standard) were quantified in real time, by fluorogenic reporter oligonucleotide probes and primers (Metabion, Munich, Germany) with the following sequences and corresponding GenBank accession numbers:* synaptophysin* (*Syp*, NM_012664) sense 5′-TTCAGGCTGCACCAAGTGTA-3′, antisense 5′-TTCAGCCGACGAGGAGTAGT-3′, probe 5′-AGGGGGCACTACCAAGATCT-3′;* neuregulin-1* (*Nrg1*, NM_001271118) sense 5′-GGGACCAGCCATCTCATAAA-3′, antisense 5′-ATCTTGACGGGTTTGACAGG-3′, probe 5′-ACTTTCTGTGTGAATGGGGG-3′;* neuropilin-1* (*Nrp1*, NM_145098) sense 5′-TGAGCCCTGTGGTCTATTCC-3′, antisense 5′-CCTCTGGCTTCTGGTAGTGC-3′, probe 5′-TGTGGGTACACTGAGGGTCA-3′; *β-actin* (*Actb*, NM_031144) sense 5′-GTACAACCTCCTTGCAGCTCCT-3′, antisense 5′-TTGTCGACGACGACGGC-3′, probe 5′-CGCCACCAGTTCGCCATGGAT-3′. Real-time PCR and detection were performed in triplicate, measurements repeated 3 times for each sample. Target gene expression was quantified according to the 2^−ΔΔCT^ method [42].

### 2.7. Statistical Analysis

Data are presented as mean + standard deviation and differences between groups were determined by one-way analysis of variance (one-way ANOVA) followed by Bonferroni post hoc test for multiple comparison with Prism 6 (GraphPad Software, La Jolla, CA, USA). For MRI results, nonparametric Mann-Whitney* U* test was used. *p* values less than 0.05 were considered as statistically significant.

The article "Erythropoietin Restores Long-Term Neurocognitive Function Involving Mechanisms of Neuronal Plasticity in a Model of Hyperoxia-Induced Preterm Brain Injury" was published in 2016. Journal: Oxid Med Cell Longev.

## 3. Results

### 3.1. Erythropoietin Attenuates Hyperoxia-Induced Long-Term Cognitive Deficits

Since neonatal exposure to hyperoxia is associated with motor-cognitive impairment in rodents [18, 19], we assessed the potential protective effect of Epo treatment on motor activity and cognitive function in adolescent (P30) and adult (P90) rats following neonatal hyperoxia (P6, 24 hours of 80% oxygen). General motor activity analysed in the open field test was affected by neither hyperoxia nor Epo treatment (Figure 1(a)). For evaluation of memory deficits we performed the novel object recognition and the Barnes maze test. For novel object recognition, the time animals spent at the familiar and novel objects was recorded. In accordance with physiological exploration behaviour [36], control animals spent significantly more time with the novel object, whereas animals in the hyperoxia group did not show preference to any object. However, upon Epo treatment we detected normalised object recognition (Figure 1(b)), suggesting that hyperoxia-induced long-term cognitive impairment can be attenuated by Epo. The exploration preference was more prominent in adolescent animals with overall reduced exploratory activity in adulthood. In the Barnes maze we found a significant increase in the latency to find the trained escape hole in adolescent as well as adult animals after neonatal hyperoxia which was absent in the Epo treated animals (Figure 1(c)). Thus, behavioural testing showed long-term cognitive impairment after neonatal hyperoxia, whereas single Epo treatment improved hyperoxia-induced memory deficits.

### 3.2. Erythropoietin Improves Oligodendrocyte Survival after Hyperoxia but Does Not Influence Hypomyelination and Long-Term Structural White Matter Injury

White matter changes have been associated with cognitive deficits of preterm born infants later in life [43] and experimental models of hyperoxia revealed striking effects on myelination and microstructural white matter changes [13, 19, 44, 45]. Since Epo application has been shown to ameliorate white matter injury [46–48], we tested whether Epo-induced restoration of cognitive function might be associated with preservation of white matter structures. To investigate the effect of hyperoxia and Epo on oligodendrocyte survival we performed immunohistochemical staining of the pan-oligodendrocyte marker Olig2 and TUNEL. We detected a significant increase in oligodendrocyte cell death at P7 after 24 hours of hyperoxia, which was significantly diminished in Epo treated animals (Figure 2(a)). To elucidate whether the preserved oligodendrocyte survival following Epo treatment was associated with protection of subacute and long-term hyperoxia-induced white matter injury we performed MBP protein expression analysis at P11 and postmortem diffusion tensor imaging (DTI) of* ex vivo* brains at P125. A significant decrease of MBP protein expression was detected in hyperoxia-exposed animals as compared to normoxic controls, which was not influenced by Epo treatment (Figure 2(b)).

The article "Erythropoietin Restores Long-Term Neurocognitive Function Involving Mechanisms of Neuronal Plasticity in a Model of Hyperoxia-Induced Preterm Brain Injury" was published in 2016. Journal: Oxid Med Cell Longev.

In accordance with MBP protein levels, fractional anisotropy (FA) as a sign of altered white matter microstructure and myelination deficit measured by DTI (Figures 3(a)–3(c)) was significantly reduced in the corpus callosum of hyperoxic animals and remained unchanged after Epo application (Figure 3(b)). The analysis of FA in the external capsule showed similar results (Figure 3(c)), although not reaching statistical significance. Of note, a single Epo injection ameliorates the neonatal hyperoxia-induced oligodendrocyte degeneration without long-lasting influence on myelination and preservation of white matter structures.

### 3.3. Hyperoxia-Induced Downregulation of Neuronal Plasticity-Associated Genes Is Ameliorated by Epo Treatment

Since Epo-induced improvement of cognitive function after neonatal hyperoxia was not directly associated with preservation of white matter structures, we investigated whether amelioration of memory deficits might be linked to changes in neuronal connectivity. We assessed mRNA expression of the synaptic plasticity-related markers* synaptophysin* (*Syp*),* neuregulin-1* (*Nrg1*), and* neuropilin-1* (*Nrp1*) 24 hours (P7) and 4 days (P11) after hyperoxia exposure and in adult animals (P125) to evaluate potential persisting effects. Interestingly, we detected significant acute (Figure 4(a)) and subacute (Figure 4(b)) downregulation of all investigated markers in hyperoxic tissue which were still prominent in adulthood (Figure 4(c)). Treatment with Epo led to significant upregulation at all investigated time points (Figures 4(a)–4(c)). Thus, hyperoxia-triggered changes in neuronal plasticity gene expression were significantly ameliorated by single Epo treatment.

## 4. Discussion

The present study demonstrates long-term cognitive improvement following Epo treatment in a neonatal rodent model of oxygen-induced brain injury. A single Epo injection at the beginning of hyperoxia (24 hours of 80% oxygen) at P6 induces oligodendrocyte preservation, however without obvious protection against hypomyelination or long-lasting microstructural white matter changes. Nevertheless, we provide clear evidence that Epo improves cognitive function which is associated with long-lasting restoration of hyperoxia-induced changes of neuronal plasticity processes.

The article "Erythropoietin Restores Long-Term Neurocognitive Function Involving Mechanisms of Neuronal Plasticity in a Model of Hyperoxia-Induced Preterm Brain Injury" was published in 2016. Journal: Oxid Med Cell Longev.

The neuroprotective effect of Epo has been widely described in experimental neonatal rodent models like hypoxia-ischemia, excitotoxicity, and stroke [27, 49]. Single-dose Epo application at the onset of 24 hours of hyperoxia was likewise repeatedly identified as neuroprotective [33, 50]. In previous studies we demonstrated that Epo mediates its protection through reduction of apoptosis, inflammation, oxidative stress responses, and modification of autophagy-associated processes [16, 32–34]. Here we show that single-dose administration of Epo significantly ameliorates oxygen-induced memory impairment in adolescence, persisting into adulthood. Whereas Barnes maze revealed similar results for both developmental stages, the exploration preference obtained by novel object recognition was more prominent in adolescent animals with generally reduced exploratory activity at the novel object in adulthood. The latter results are in accordance with Stansfield and Kirstein describing adolescent animals spending more time with a novel object relative to adults [51]. Epo's cognitive improvement properties have also been found in other neonatal injury models, that is, neonatal stroke/hypoxia-ischemia, which revealed a long-term improved neurological outcome after Epo treatment [52, 53]. It has been shown that the neuroprotective dose in animal models is much higher than the one used for support of erythropoiesis in the newborn [54]. This is further supported by reports in other experimental neonatal brain injury models, that is, hypoxia-ischemia. Here it was shown that that plasma concentrations shown to be neuroprotective in seven-day-old rats receiving 5000 IU/kg equal those obtained by 1000 IU/kg Epo per dose in term infants. These studies suggest that higher doses need to be administered in rats compared to humans [55, 56]. The Epo dose in the present work was chosen according to our own previous studies and based on the literature with numerous experimental evidences of neuroprotection in six-day-old rats [16, 32–34, 50].

In the clinical setting, several safety studies revealed a good tolerance for high Epo doses administered to preterm infants [48, 54, 55, 57–59]. Follow-up of patients included in these studies as well as first clinical trials designed to investigate neurological outcome after Epo treatment indicated that cognitive performance is improved up to the age of four years. However, these trials differed in design and dose of Epo used: Mcadams et al. did a retrospective analysis of the neurodevelopmental outcome of 60 patients included in a pharmacokinetic trial evaluating the effects of high-dose Epo over a short period of time. Ohls and coworkers aimed at investigating the difference between chronic application of low-dose Epo and Darbepoetin on the outcome in preschool age [60–62]. Since further investigation of the adolescent and adult developmental outcome will take decades in the clinic, our data provide first evidence for a long-lasting neuroprotective effect of Epo on the cognitive outcome in a preterm model of brain injury.

The article "Erythropoietin Restores Long-Term Neurocognitive Function Involving Mechanisms of Neuronal Plasticity in a Model of Hyperoxia-Induced Preterm Brain Injury" was published in 2016. Journal: Oxid Med Cell Longev.

Although there is an increased understanding regarding the neuroprotective mode of action of Epo in experimental models of neonatal brain injury, the underlying mechanisms are not completely understood and may differ between models. One aim of this study was to investigate the possible impact of Epo on white matter preservation. In general, the phase of greatest vulnerability of the developing brain coincides with the peak of the brain growth spurt, in humans starting at mid-pregnancy and extending into the third year of life. Rodents show a delay in brain maturation and myelination, starting in the first postnatal days of life and therefore corresponding to immature born infants (23–36 weeks of gestation) [63, 64]. In preterms, the leading cause of motor and cognitive disturbances in later life consists of cerebral grey and white matter injuries [65]. Particularly, microstructural abnormalities in particular white matter regions are related to long-lasting impairment [66]. Previous experimental studies revealed that neonatal hyperoxia-triggered neural cell degeneration leads to a transient hypomyelination with disrupted axon-oligodendrocyte integrity and long-lasting microstructural changes in white matter up to the fully adult developmental stage [11, 13, 14, 19, 44, 45, 67, 68]. The present study shows that a single Epo application significantly decreases oligodendrocyte cell death in the developing brain following neonatal hyperoxia. Interestingly, there is no protection from hypomyelination. The absence of a protective effect differs from findings in other injury models of the mature and immature brain, where systemic Epo application induced an increased proliferation and differentiation of oligodendrocyte progenitor cells as well as preservation of the white matter [47, 69–72]. Even chronic Epo administration over a period of three weeks in healthy young mice was shown to increase the number and differentiation of neural cells without increased proliferation or decreased cell degeneration [73]. The majority of studies did not investigate changes up to the adult developmental stage, leaving long-term myelination partially undefined. Our data reveal hyperoxia-induced changes in white matter microstructures on diffusion tensor imaging, that is, reduced fractional anisotropy of adult rat brains, which are likewise not restored by Epo treatment. These findings differ from clinical trials, where Epo-mediated protection improved white matter integrity assessed by MRI in preterm infants [48, 59]. However, imaging was performed at term equivalent age and therefore at a different developmental stage in comparison to our study. Keeping the complex phenotype and the multiple origins of pathology of preterm infants in mind, limitations of our single-hit experimental model have to be taken into account. In contrast to the present work, other studies applied different Epo treatment regimes, using chronic applications of lower dosage instead of single high-dose treatment. Our data suggest that single Epo administration leads to protection of degenerating oligodendrocytes after neonatal hyperoxia. However, in addition to oligodendrocyte cell death hyperoxia also alters differentiation and maturation [13, 19, 44, 45, 67], which have not been investigated on a cellular level in the current study. Thus, it cannot be excluded that the lack of myelin-preservation might have been caused by insufficient promotion of differentiation by single-dose usage of Epo, possibly resulting in a reduced number of myelin-producing, mature oligodendrocytes. Therefore, a multiple-dose treatment regime should be investigated in further studies to elucidate additional cellular effects regarding white matter development.

The article "Erythropoietin Restores Long-Term Neurocognitive Function Involving Mechanisms of Neuronal Plasticity in a Model of Hyperoxia-Induced Preterm Brain Injury" was published in 2016. Journal: Oxid Med Cell Longev.

The detrimental effect of neonatal hyperoxia on neuronal survival and differentiation has been described previously [74–76]. It has been further shown that Epo protects neurons from degeneration in different disease models of the mature and immature brain [53, 77, 78]. The impact of hyperoxia with and without application of Epo on neuronal plasticity, however, has not been addressed so far. Synaptic plasticity is the ability of synapses to modify transmission in strength or efficacy. Changes in synaptic plasticity have been reported to play a critical role in memory formation. In addition to the key effector mechanisms of Epo associated with neuroprotection, high expression of the Epo receptor on cortical and hippocampal neurons has been related to higher synaptic plasticity and cognitive performance [79]. Moreover, administration of Epo decreases the excitatory neurotransmitter release probability, enhances synaptic plasticity in mice hippocampal slices, and improves hippocampus dependent memory by modulating plasticity, synaptic connectivity, and activity of memory-related neuronal networks [80, 81]. To investigate the effect of hyperoxia and Epo application on neuronal plasticity we assessed mRNA expression of the associated markers* synaptophysin* (*Syp*),* neuregulin-1* (*Nrg1*), and* neuropilin-1* (*Nrp1*).* Synaptophysin* is an integral synaptic vesicle protein considered to be a representative for synaptic density and synaptogenesis [82].* Neuregulin-1*, a member of the epidermal growth factor family, shows high affinity to ErbB4 receptor, whereas Nrg1-ErbB4 signalling has been described to play a critical role in neurotransmission, synaptic plasticity, and synchronisation of neuronal network activity [83–85].* Neuropilin-1*, a transmembrane protein receptor, is supposed to be important for axon patterning of motor and sensory nerves after binding to* semaphorin-3A* [86]. Our data indicate that the protective effects of single-dose Epo administration are linked to changes in neuronal plasticity. These findings are in accordance with increasing evidence suggesting that age-related decreases of Epo expression in the hippocampal region may contribute to Alzheimer (AD), a disease well known to be associated with neurodegeneration and apoptosis which impair synaptic function [87–90]. Moreover, in adult injury models of AD, administration of Epo has been shown to improve synaptic plasticity and memory deficits which were associated with increased cerebral synaptophysin expression [91, 92]. After rodent spinal cord injury, injection of nonreplicating herpes simplex virus based vector coding for Epo also improved the functional outcome and increased synaptic proteins synaptophysin and postsynaptic density protein-95 [93]. Therefore, Epo-mediated regulation of synaptic plasticity genes may be one effector mechanism to improve the cognitive outcome after neonatal brain injury. Further studies will be required to unravel the detailed molecular mechanisms underlying the observed regulation of Epo-mediated alterations in plasticity-related gene expression.

The article "Erythropoietin Restores Long-Term Neurocognitive Function Involving Mechanisms of Neuronal Plasticity in a Model of Hyperoxia-Induced Preterm Brain Injury" was published in 2016. Journal: Oxid Med Cell Longev.

## 5. Conclusion

In summary, our study reveals that administration of Epo in oxygen-induced brain injury leads to an improved cognitive outcome. Analysis of neuronal plasticity markers demonstrates a hyperoxia-triggered persistent downregulation, which can be reversed by Epo treatment. Therefore, changes in plasticity processes might contribute to an ameliorated neurocognitive outcome.

These findings are highly relevant from a clinical perspective since oxygen administration in neonates is sometimes inevitable and premature infants are already exposed to oxygen concentrations after birth fourfold higher compared to intrauterine conditions. Therefore, any therapy needs to be applied immediately at the onset of hyperoxia. To support the very vulnerable phase of brain maturation and enhance the developmental and regenerative potential of the preterm brain, it is crucial to investigate safe treatment options, like erythropoietin, to better understand the underlying molecular and cellular mechanisms and facilitate transition into the clinical setting. In conclusion, our results underline once more the importance of Epo as a candidate for neuroprotective therapy in neonates.

## Figures and Tables

**Figure 1:** Erythropoietin improved cognitive function following neonatal hyperoxia. Motor-cognitive development was assessed by open field, novel object recognition, and Barnes maze starting at P30 (adolescent) and P90 (adult) after exposure to neonatal normoxia (21% oxygen (21%)) or hyperoxia (24 h, 80% oxygen (80%)) at P6 combined with i.p. administration of normal saline or 20,000 IU/kg Epo. (a) To test general motor activity animals were placed into the open field maze for 10 minutes. Movement of animals was tracked automatically by the software through three-point detection and the centre of the animals was analysed. Motor activity was expressed by the mean velocity and the total distance. (b) Cognitive function was assessed in the novel object recognition task presented as the exploration time at the novel object (N) versus familiar objects (F1 and F2). (c) Memory function was determined in the Barnes maze test expressed as the latency to find the trained escape hole after a 3-day training period. *n* = 8–10 rats/group. ^*∗*^ *p* < 0.05, ^*∗∗*^ *p* < 0.01, and ^*∗∗∗*^ *p* < 0.001.

**Figure 2:** Erythropoietin ameliorates oligodendrocyte degeneration but not hyperoxia-mediated hypomyelination. (a) Oligodendrocyte degeneration was determined in brain sections from P7 rats that were exposed to either normoxia (21% oxygen (21%)) or hyperoxia (24 h, 80% oxygen (80%)) at P6 and treated with normal saline or 20,000 IU/kg Epo. Oligodendrocyte degeneration was determined by immunohistochemical TUNEL (green)/Olig2 (red) and DAPI (not depicted) costaining (positive counted cells appear yellow and are marked by arrows). Scale  bar = 50 *μ*m, *n* = 8–10 rats/group. (b) Myelin basic protein (MBP) expression was analysed 4 days after hyperoxia in protein lysates of complete hemispheres (excluding cerebellum). *n* = 8–10 rats/group. ^*∗∗*^ *p* < 0.01, ^*∗∗∗*^ *p* < 0.001.

**Figure 3:** Long-term white matter microstructural development is not improved by a single injection of erythropoietin. (a) Representative T_2_W images (b_0_), fractional anisotropy (FA) maps, and direction encoded colour maps (DEC) of a P125 control rat (21%) derived from diffusion tensor imaging showing the different levels used for quantitative analysis. Corpus callosum (CC) and external capsule (EC) are displayed on the DEC. Diffusivity values of radial diffusivity (*D*_⊥_), axial diffusivity (*D*_//_), mean diffusivity (MD), and fractional anisotropy in corpus callosum (b) and external capsule (c) determined by diffusion tensor imaging out of rats exposed to normoxia (21% oxygen (21%)) or hyperoxia (24 h, 80% oxygen (80%)) at P6 and treated with normal saline or 20,000 IU/kg Epo. *n* = 6 rats/group. ^*∗*^ *p* < 0.05, ^*∗∗*^ *p* < 0.01.

The article "Erythropoietin Restores Long-Term Neurocognitive Function Involving Mechanisms of Neuronal Plasticity in a Model of Hyperoxia-Induced Preterm Brain Injury" was published in 2016. Journal: Oxid Med Cell Longev.

**Figure 4:** Erythropoietin restores plasticity-related genes following neonatal hyperoxia.* Synaptophysin* (*Syp*),* neuregulin-1* (*Nrg1*), and* neuropilin-1* (*Nrp1*) mRNA expression in hemispheres of (a) P7, (b) P11, and (c) P125 rats exposed to either normoxia (21% oxygen (21%)) or hyperoxia (24 h, 80% oxygen (80%)) at P6 and treated with normal saline or 20,000 IU/kg Epo i.p. *n* = 4–8 rats/group. ^*∗*^ *p* < 0.05, ^*∗∗*^ *p* < 0.01, and ^*∗∗∗*^ *p* < 0.001.

## References

[1] Wilson-Costello D., Friedman H., Minich N., Fanaroff A. A., Hack M. (2005). Improved survival rates with increased neurodevelopmental disability for extremely low birth weight infants in the 1990s. *Pediatrics*.

[2] Platt M. J., Cans C., Johnson A. (2007). Trends in cerebral palsy among infants of very low birthweight (<1500 g) or born prematurely (<32 weeks) in 16 European centres: a database study. *The Lancet*.

[3] Sellier E., Platt M. J., Andersen G. L., Krägeloh-Mann I., De La Cruz J., Cans C. (2016). Decreasing prevalence in cerebral palsy: a multi-site European population-based study, 1980 to 2003. *Developmental Medicine & Child Neurology*.

[4] Pavlova M. A., Krägeloh-Mann I. (2013). Limitations on the developing preterm brain: impact of periventricular white matter lesions on brain connectivity and cognition. *Brain*.

[5] Dean J. M., Bennet L., Back S. A., McClendon E., Riddle A., Gunn A. J. (2014). What brakes the preterm brain? An arresting story. *Pediatric Research*.

[6] Anderson P. J., De Luca C. R., Hutchinson E. (2011). Attention problems in a representative sample of extremely preterm/extremely low birth weight children. *Developmental Neuropsychology*.

[7] Anderson P. J., Doyle L. W. (2008). Cognitive and Educational Deficits in Children Born Extremely Preterm. *Seminars in Perinatology*.

[8] Collins M. P., Lorenz J. M., Jetton J. R., Paneth N. (2001). Hypocapnia and other ventilation-related risk factors for cerebral palsy in low birth weight infants. *Pediatric Research*.

[9] Rabi Y., Rabi D., Yee W. (2007). Room air resuscitation of the depressed newborn: a systematic review and meta-analysis. *Resuscitation*.

The article "Erythropoietin Restores Long-Term Neurocognitive Function Involving Mechanisms of Neuronal Plasticity in a Model of Hyperoxia-Induced Preterm Brain Injury" was published in 2016. Journal: Oxid Med Cell Longev.

[10] Saugstad O. D., Ramji S., Soll R. F., Vento M. (2008). Resuscitation of newborn infants with 21% or 100% oxygen: an updated systematic review and meta-analysis. *Neonatology*.

[11] Felderhoff-Mueser U., Bittigau P., Sifringer M. (2004). Oxygen causes cell death in the developing brain. *Neurobiology of Disease*.

[12] Sirinyan M., Sennlaub F., Dorfman A. (2006). Hyperoxic exposure leads to nitrative stress and ensuing microvascular degeneration and diminished brain mass and function in the immature subject. *Stroke*.

[13] Brehmer F., Bendix I., Prager S. (2012). Interaction of inflammation and hyperoxia in a rat model of neonatal white matter damage. *PLoS ONE*.

[14] Dzietko M., Boos V., Sifringer M. (2008). A critical role for Fas/CD-95 dependent signaling pathways in the pathogenesis of hyperoxia-induced brain injury. *Annals of Neurology*.

[15] Gerstner B., DeSilva T. M., Genz K. (2008). Hyperoxia causes maturation-dependent cell death in the developing white matter. *The Journal of Neuroscience*.

[16] Sifringer M., Genz K., Brait D. (2009). Erythropoietin attenuates hyperoxia-induced cell death by modulation of inflammatory mediators and matrix metalloproteinases. *Developmental Neuroscience*.

[17] Vottier G., Pham H., Pansiot J. (2011). Deleterious effect of hyperoxia at birth on white matter damage in the newborn rat. *Developmental Neuroscience*.

[18] Schmitz T., Endesfelder S., Reinert M.-C. (2012). Adolescent hyperactivity and impaired coordination after neonatal hyperoxia. *Experimental Neurology*.

[19] Serdar M., Herz J., Kempe K. (2016). Fingolimod protects against neonatal white matter damage and long-term cognitive deficits caused by hyperoxia. *Brain, Behavior, and Immunity*.

[20] Maier R. F., Obladen M., Scigalla P. (1994). The effect of epoetin beta (recombinant human erythropoietin) on the need for transfusion in very-low-birth-weight infants. *The New England Journal of Medicine*.

[21] Neubauer A.-P., Voss W., Wachtendorf M., Jungmann T. (2010). Erythropoietin improves neurodevelopmental outcome of extremely preterm infants. *Annals of Neurology*.

[22] Chen Z.-Y., Asavaritikrai P., Prchal J. T., Noguchi C. T. (2007). Endogenous erythropoietin signaling is required for normal neural progenitor cell proliferation. *Journal of Biological Chemistry*.

[23] Sakanaka M., Wen T.-C., Matsuda S. (1998). *In vivo* evidence that erythropoietin protects neurons from ischemic damage. *Proceedings of the National Academy of Sciences of the United States of America*.

[24] Fan X., van Bel F., van der Kooij M. A., Heijnen C. J., Groenendaal F. (2013). Hypothermia and erythropoietin for neuroprotection after neonatal brain damage. *Pediatric Research*.

The article "Erythropoietin Restores Long-Term Neurocognitive Function Involving Mechanisms of Neuronal Plasticity in a Model of Hyperoxia-Induced Preterm Brain Injury" was published in 2016. Journal: Oxid Med Cell Longev.

[25] Gonzalez F. F., Larpthaveesarp A., McQuillen P. (2013). Erythropoietin Increases neurogenesis and oligodendrogliosis of subventricular zone precursor cells after neonatal stroke. *Stroke*.

[26] Traudt C. M., McPherson R. J., Bauer L. A. (2013). Concurrent erythropoietin and hypothermia treatment improve outcomes in a term nonhuman primate model of perinatal asphyxia. *Developmental Neuroscience*.

[27] Juul S. E., Pet G. C. (2015). Erythropoietin and Neonatal Neuroprotection. *Clinics in Perinatology*.

[28] Jantzie L. L., Corbett C. J., Berglass J. (2014). Complex pattern of interaction between in utero hypoxia-ischemia and intra-amniotic inflammation disrupts brain development and motor function. *Journal of Neuroinflammation*.

[29] Jantzie L. L., Corbett C. J., Firl D. J., Robinson S. (2015). Postnatal erythropoietin mitigates impaired cerebral cortical development following subplate loss from prenatal hypoxia-ischemia. *Cerebral Cortex*.

[30] van de Looij Y., Chatagner A., Quairiaux C., Gruetter R., Hüppi P. S., Sizonenko S. V. (2014). Multi-modal assessment of long-term erythropoietin treatment after neonatal hypoxic-ischemic injury in rat brain. *PLoS ONE*.

[31] Back S. A., Rosenberg P. A. (2014). Pathophysiology of glia in perinatal white matter injury. *Glia*.

[32] Bendix I., Schulze C., von Haefen C. (2012). Erythropoietin modulates autophagy signaling in the developing rat brain in an in vivo model of Oxygen-Toxicity. *International Journal of Molecular Sciences*.

[33] Kaindl A. M., Sifringer M., Koppelstaetter A. (2008). Erythropoietin protects the developing brain from hyperoxia-induced cell death and proteome changes. *Annals of Neurology*.

[34] Sifringer M., Brait D., Weichelt U. (2010). Erythropoietin attenuates hyperoxia-induced oxidative stress in the developing rat brain. *Brain, Behavior, and Immunity*.

[35] Defries J. C., Hegmann J. P., Weir M. W. (1966). Open-field behavior in mice: evidence for a major gene effect mediated by the visual system. *Science*.

[36] Chambon C., Wegener N., Gravius A., Danysz W. (2011). A new automated method to assess the rat recognition memory: validation of the method. *Behavioural Brain Research*.

[37] Barnes C. A. (1979). Memory deficits associated with senescence: a neurophysiological and behavioral study in the rat. *Journal of Comparative and Physiological Psychology*.

[38] O'Leary T. P., Savoie V., Brown R. E. (2011). Learning, memory and search strategies of inbred mouse strains with different visual abilities in the Barnes maze. *Behavioural Brain Research*.

[39] Harauz G., Boggs J. M. (2013). Myelin management by the 18.5-kDa and 21.5-kDa classic myelin basic protein isoforms. *Journal of Neurochemistry*.

The article "Erythropoietin Restores Long-Term Neurocognitive Function Involving Mechanisms of Neuronal Plasticity in a Model of Hyperoxia-Induced Preterm Brain Injury" was published in 2016. Journal: Oxid Med Cell Longev.

[40] Basser P. J., Pierpaoli C. (1998). A simplified method to measure the diffusion tensor from seven MR images. *Magnetic Resonance in Medicine*.

[41] Sifringer M., Bendix I., von Haefen C. (2013). Oxygen toxicity is reduced by acetylcholinesterase inhibition in the developing rat brain. *Developmental Neuroscience*.

[42] Livak K. J., Schmittgen T. D. (2001). Analysis of relative gene expression data using real-time quantitative PCR and the 2-ΔΔCT method. *Methods*.

[43] Soria-Pastor S., Gimenez M., Narberhaus A. (2008). Patterns of cerebral white matter damage and cognitive impairment in adolescents born very preterm. *International Journal of Developmental Neuroscience*.

[44] Ritter J., Schmitz T., Chew L.-J. (2013). Neonatal hyperoxia exposure disrupts axon-oligodendrocyte integrity in the subcortical white matter. *The Journal of Neuroscience*.

[45] Schmitz T., Krabbe G., Weikert G. (2014). Minocycline protects the immature white matter against hyperoxia. *Experimental Neurology*.

[46] Iwai M., Stetler R. A., Xing J. (2010). Enhanced oligodendrogenesis and recovery of neurological function by erythropoietin after neonatal hypoxic/ischemic brain injury. *Stroke*.

[47] Kako E., Kaneko N., Aoyama M. (2012). Subventricular zone-derived oligodendrogenesis in injured neonatal white matter in mice enhanced by a nonerythropoietic erythropoietin derivative. *Stem Cells*.

[48] O'Gorman R. L., Bucher H. U., Held U. (2015). Tract-based spatial statistics to assess the neuroprotective effect of early erythropoietin on white matter development in preterm infants. *Brain*.

[49] Juul S., Felderhoff-Mueser U. (2007). Epo and other hematopoietic factors. *Seminars in Fetal and Neonatal Medicine*.

[50] Yiş U., Kurul S. H., Kumral A. (2008). Effect of erythropoietin on oxygen-induced brain injury in the newborn rat. *Neuroscience Letters*.

[51] Stansfield K. H., Kirstein C. L. (2006). Effects of novelty on behavior in the adolescent and adult rat. *Developmental Psychobiology*.

[52] Demers E. J., McPherson R. J., Juul S. E. (2005). Erythropoietin protects dopaminergic neurons and improves neurobehavioral outcomes in juvenile rats after neonatal hypoxia-ischemia. *Pediatric Research*.

[53] Lan K. M., Tien L. T., Cai Z. (2016). Erythropoietin ameliorates neonatal hypoxia-ischemia-induced neurobehavioral deficits, neuroinflammation, and hippocampal injury in the Juvenile rat. *International Journal of Molecular Sciences*.

[54] Kellert B. A., McPherson R. J., Juul S. E. (2007). A comparison of high-dose recombinant erythropoietin treatment regimens in brain-injured neonatal rats. *Pediatric Research*.

The article "Erythropoietin Restores Long-Term Neurocognitive Function Involving Mechanisms of Neuronal Plasticity in a Model of Hyperoxia-Induced Preterm Brain Injury" was published in 2016. Journal: Oxid Med Cell Longev.

[55] Statler P. A., Mcpherson R. J., Bauer L. A., Kellert B. A., Juul S. E. (2007). Pharmacokinetics of high-dose recombinant erythropoietin in plasma and brain of neonatal rats. *Pediatric Research*.

[56] Wu Y. W., Bauer L. A., Ballard R. A. (2012). Erythropoietin for neuroprotection in neonatal encephalopathy: safety and pharmacokinetics. *Pediatrics*.

[57] Fauchère J.-C., Dame C., Vonthein R. (2008). An approach to using recombinant erythropoietin for neuroprotection in very preterm infants. *Pediatrics*.

[58] Juul S. E., McPherson R. J., Bauer L. A., Ledbetter K. J., Gleason C. A., Mayock D. E. (2008). A phase I/II trial of high-dose erythropoietin in extremely low birth weight infants: pharmacokinetics and safety. *Pediatrics*.

[59] Leuchter R. H.-V., Gui L., Poncet A. (2014). Association between early administration of high-dose erythropoietin in preterm infants and brain MRI abnormality at term-equivalent age. *The Journal of the American Medical Association*.

[60] Mcadams R. M., Mcpherson R. J., Mayock D. E., Juul S. E. (2013). Outcomes of extremely low birth weight infants given early high-dose erythropoietin. *Journal of Perinatology*.

[61] Ohls R. K., Cannon D. C., Phillips J. (2016). Preschool assessment of preterm infants treated with darbepoetin and erythropoietin. *Pediatrics*.

[62] Ohls R. K., Kamath-Rayne B. D., Christensen R. D. (2014). Cognitive outcomes of preterm infants randomized to darbepoetin, erythropoietin, or placebo. *Pediatrics*.

[63] Dobbing J., Sands J. (1979). Comparative aspects of the brain growth spurt. *Early Human Development*.

[64] Semple B. D., Blomgren K., Gimlin K., Ferriero D. M., Noble-Haeusslein L. J. (2013). Brain development in rodents and humans: identifying benchmarks of maturation and vulnerability to injury across species. *Progress in Neurobiology*.

[65] Volpe J. J. (2009). Brain injury in premature infants: a complex amalgam of destructive and developmental disturbances. *The Lancet Neurology*.

[66] Counsell S. J., Edwards A. D., Chew A. T. M. (2008). Specific relations between neurodevelopmental abilities and white matter microstructure in children born preterm. *Brain*.

[67] Schmitz T., Ritter J., Mueller S., Felderhoff-Mueser U., Chew L.-J., Gallo V. (2011). Cellular changes underlying hyperoxia-induced delay of white matter development. *Journal of Neuroscience*.

[68] Sifringer M., Bendix I., Börner C. (2012). Prevention of neonatal oxygen-induced brain damage by reduction of intrinsic apoptosis. *Cell Death and Disease*.

[69] Cho Y. K., Kim G., Park S. (2012). Erythropoietin promotes oligodendrogenesis and myelin repair following lysolecithin-induced injury in spinal cord slice culture. *Biochemical and Biophysical Research Communications*.

The article "Erythropoietin Restores Long-Term Neurocognitive Function Involving Mechanisms of Neuronal Plasticity in a Model of Hyperoxia-Induced Preterm Brain Injury" was published in 2016. Journal: Oxid Med Cell Longev.

[70] Fan X., Heijnen C. J., Van Der Kooij M. A., Groenendaal F., Van Bel F. (2011). Beneficial effect of erythropoietin on sensorimotor function and white matter after hypoxia-ischemia in neonatal mice. *Pediatric Research*.

[71] Kaneko N., Kako E., Sawamoto K. (2013). Enhancement of ventricular-subventricular zone-derived neurogenesis and oligodendrogenesis by erythropoietin and its derivatives. *Frontiers in Cellular Neuroscience*.

[72] Zhang L., Chopp M., Zhang R. L. (2010). Erythropoietin amplifies stroke-induced oligodendrogenesis in the rat. *PLoS ONE*.

[73] Hassouna I., Ott C., Wüstefeld L. (2016). Revisiting adult neurogenesis and the role of erythropoietin for neuronal and oligodendroglial differentiation in the hippocampus. *Molecular Psychiatry*.

[74] Endesfelder S., Zaak I., Weichelt U., Bührer C., Schmitz T. (2014). Caffeine protects neuronal cells against injury caused by hyperoxia in the immature brain. *Free Radical Biology and Medicine*.

[75] Liu Y., Jiang P., Du M. (2015). Hyperoxia-induced immature brain injury through the TLR4 signaling pathway in newborn mice. *Brain Research*.

[76] Topçu Y., Bayram E., Özbal S. (2014). Zonisamide attenuates hyperoxia-induced apoptosis in the developing rat brain. *Neurological Sciences*.

[77] Liu X.-B., Wang J.-A., Yu S. P., Keogh C. L., Wei L. (2008). Therapeutic strategy for erythropoietin in neurological disorders. *CNS and Neurological Disorders—Drug Targets*.

[78] Osredkar D., Sall J. W., Bickler P. E., Ferriero D. M. (2010). Erythropoietin promotes hippocampal neurogenesis in in vitro models of neonatal stroke. *Neurobiology of Disease*.

[79] Sargin D., El-Kordi A., Agarwal A. (2011). Expression of constitutively active erythropoietin receptor in pyramidal neurons of cortex and hippocampus boosts higher cognitive functions in mice. *BMC Biology*.

[80] Adamcio B., Sargin D., Stradomska A. (2008). Erythropoietin enhances hippocampal long-term potentiation and memory. *BMC Biology*.

[81] Kamal A., Al Shaibani T., Ramakers G. (2011). Erythropoietin decreases the excitatory neurotransmitter release probability and enhances synaptic plasticity in mice hippocampal slices. *Brain Research*.

[82] Eastwood S. L., Weickert C. S., Webster M. J., Herman M. M., Kleinman J. E., Harrison P. J. (2006). Synaptophysin protein and mRNA expression in the human hippocampal formation from birth to old age. *Hippocampus*.

[83] Eto K., Hommyo A., Yonemitsu R., Abe S.-I. (2010). ErbB4 signals Neuregulin1-stimulated cell proliferation and c-fos gene expression through phosphorylation of serum response factor by mitogen-activated protein kinase cascade. *Molecular and Cellular Biochemistry*.

The article "Erythropoietin Restores Long-Term Neurocognitive Function Involving Mechanisms of Neuronal Plasticity in a Model of Hyperoxia-Induced Preterm Brain Injury" was published in 2016. Journal: Oxid Med Cell Longev.

[84] Fisahn A., Neddens J., Yan L., Buonanno A. (2009). Neuregulin-1 modulates hippocampal gamma oscillations: implications for schizophrenia. *Cerebral Cortex*.

[85] Mei L., Xiong W.-C. (2008). Neuregulin 1 in neural development, synaptic plasticity and schizophrenia. *Nature Reviews Neuroscience*.

[86] Fantin A., Maden C. H., Ruhrberg C. (2009). Neuropilin ligands in vascular and neuronal patterning. *Biochemical Society Transactions*.

[87] Chung Y. H., Kim S. I., Joo K. M. (2004). Age-related changes in erythropoietin immunoreactivity in the cerebral cortex and hippocampus of rats. *Brain Research*.

[88] Kuang X., Du J.-R., Chen Y.-S., Wang J., Wang Y.-N. (2009). Protective effect of Z-ligustilide against amyloid *β*-induced neurotoxicity is associated with decreased pro-inflammatory markers in rat brains. *Pharmacology Biochemistry and Behavior*.

[89] Shankar G. M., Li S., Mehta T. H. (2008). Amyloid-*β* protein dimers isolated directly from Alzheimer's brains impair synaptic plasticity and memory. *Nature Medicine*.

[90] Tackenberg C., Grinschgl S., Trutzel A. (2013). NMDA receptor subunit composition determines beta-amyloid-induced neurodegeneration and synaptic loss. *Cell Death and Disease*.

[91] Esmaeili Tazangi P., Moosavi S. M. S., Shabani M., Haghani M. (2015). Erythropoietin improves synaptic plasticity and memory deficits by decrease of the neurotransmitter release probability in the rat model of Alzheimer's disease. *Pharmacology Biochemistry and Behavior*.

[92] Lee S.-T., Chu K., Park J.-E. (2012). Erythropoietin improves memory function with reducing endothelial dysfunction and amyloid-beta burden in Alzheimer's disease models. *Journal of Neurochemistry*.

[93] Wang S., Wu Z., Chiang P. P., Fink D. J., Mata M. (2012). Vector-mediated expression of erythropoietin improves functional outcome after cervical spinal cord contusion injury. *Gene Therapy*.

